# Prevalence and determinants of modern contraceptive utilization among women in the reproductive age group in Edaga-hamus Town, Eastern zone, Tigray region, Ethiopia, June 2017

**DOI:** 10.1371/journal.pone.0227795

**Published:** 2020-03-06

**Authors:** Desta Tukue, Teferi Gebru Gebremeskel, Lemlem Gebremariam, Bereket Aregawi, Merhawit Gebremeskel Hagos, Tsega Gebremichael, Haben Nuguse Tesfay, Zekarias Gessesse Arefaine

**Affiliations:** 1 Obstetrician and Gynecologist in Adigrat General Hospital, Adigrat, Ethiopia; 2 Department of Reproductive Health, College of Health Sciences, Aksum University, Aksum, Ethiopia; 3 Department of Public Health, College of Medicine and Health Science, Adigrat University, Adigrat, Ethiopia; 4 Department of Internal Medicine Department, Collage of Medicine and Health Science, Aksum University, Aksum, Ethiopia; 5 Department of Midwifery, College of Medicine and Health Sciences, Aksum University, Aksum, Ethiopia; 6 Department of Epidemiology and Bioststistics, College of Medicine and Health Sciences, Aksum University, Aksum, Ethiopia; 7 Department of Pedatrics, College of Medicine and Health Sciences, Aksum University, Aksum, Ethiopia; 8 Department of Internal Medicine, College of Medicine and Health Sciences, Mekelle University, Mekelle, Ethiopia; University of Gondar, ETHIOPIA

## Abstract

**Introduction:**

All individuals and couples have a basic human right to decide freely and responsibly the number, spacing, and timing of their child. However, In Ethiopia, the prevalence of contraceptive utilization remains low and it varies in different regions. Therefore, this study was aimed to determine prevalence and determinant factors affecting the utilization of modern contraception in the reproductive age group (15–49 years) in Edaga-Hamus Town.

**Methodology:**

A community based Cross-Sectional study was carried out on April 23 to May 10, 2017. A systemic random sampling method was used to select study participants. Information was collected using a structured, pre-tested questionnaire. The data were entered into EPI-info version 7.1 and imported to SPSS version 20. Summary statistics and logistic regression analysis were performed using SPSS version 20. Those variables having a P-value of less than 0.2 in the bivariable analysis were fitted in multivariable analysis. AOR with 95% CI and P-value<0.05 were used during multivariable analysis to identify the factors associated with the utilization of modern in reproductive.

**Result:**

In this study the overall prevalence of modern contraceptive utilization was 58.5%. Age (AOR = 0.406,95%,Cl: (0.000,0.398)), Educational status (AOR = 0.901,95% Cl (0.340,4.107)), Feeling of husband towards Modern contraceptive (AOR = 0.186, 95% CI (0.056,0.617) had protective effect of utilization of modern contraceptive. But Number of children 1–3 and 4–5 wanted(AOR = 10.802,95%(4.027,28.975)), AOR = 2.624,95% CI (1.437,4.791), was a risk for utilization of modern contraceptive.

**Conclusion and recommendation:**

The prevalence of Modern contraceptive utilization was still to be low (far below the national target). Therefore, providing educational opportunities, creating awareness about contraception and effective counseling would increase modern contraceptive methods utilization.

## Introduction

According to the world health organization world statistics report, trends of maternal mortality rate are reduced from 385 to 216 globally, 538 to 176 in South Asia, 987 to 546 in sub-Saharan Africa and 1250 to 353 in Ethiopia from 1990 to 2015[1]. In developing regions the overall MMR is 239, which is nearly 20 times higher than that of developed regions[1]. Sub-Saharan Africa takes a very high maternal mortality rate[2]. Ethiopian Ministry of health has taken different types of an initiative to decrease maternal morbidity and mortality, like accessing Modern family planning service at health facilities throughout the country since 1980. According to the United Nations, official population estimates and projections in 2050 the world population will be in the range of 7.3 billion to 10.7 billion persons. About 96% of the total annual population increase occurs in less developed regions[2,3]. Around the world, about 222 million women have an unmet need for family planning and 645 million women have their needs met through the use of a modern contraceptive method, nine children under age 5 die in Africa which resulted in the death of 4.8 million children annually[4]. Sub Saharan Africa faces the most serious population and reproductive health challenges including the highest maternal mortality, population growth rate, total fertility rate and much unmet need for family planning in the world. Ethiopia is considered to be one of the most populous countries in Africa; only less than 23% of women in the reproductive age group are currently using contraception, which is still low to affect fertility following Nigeria and Egypt[5].

Modern contraceptive use by currently married Ethiopian women has steadily increased over the last 15 years, jumping from 6% of women using modern contraceptive method in 2000 to 35% in 2016, and the largest growth has been in injectables use, which expanded from use by 3% of women in 2000 to 23% in 2016, followed by growth in implant use, from less than 1% of women using in 2000 to 8% in 2016[6]. This has resulted in high rates of unwanted pregnancies, unplanned deliveries and unsafe abortions resulting in high maternal mortalities in the regions [2, 7–9].

In Ethiopia there is regional variation in modern contraceptive utilization; in Somali (1%), Afar (12%), Oromiya (28%), Benishangul-Gumuz(28%), Dire Dawa(29) Harari(29%) Gambela(35%), Tigray(35%), SNNPR(40%), Amhara(47%) Addis Ababa(50%)[6].

Study conduct in Ofla District, Tigray, Northern Ethiopia (37.1%)[10], in Tigray, North Ethiopia(35.6%)[11], in Humera town, Tigray Region, Ethiopia(27.1%)[12], in Tigray, Ethiopia(46%)[13], Addis Ababa (56.3%)[14], Debre Birhan district North Showa zone, central Ethiopia (46.9%)[15], Tigray region (32.5%)[16] and in Gondar town, northwest Ethiopia reported contraceptive utilization of 48.4 respectively[17].

Studies conducted in the Tigray region and other parts of Ethiopia showed factors found to be associated with the utilization of contraceptives vary. These include educational level, socio-cultural beliefs and practices, level of knowledge, myths, fear of side effects, partner's objection, convenience, fertility intentions, accessibility, providers' skill and competence, and other factors in the service area. These factors go a long way to influence the type of contraceptive one decides to use and use[18]. The finding of the mini EDHS 2016 (a UMC of 35.5%) for the Tigray region was striking and found to be lower than the UMC of other big regions of Ethiopia. Tigray region was believed to be one of the best performing regions as regards family planning service provision however the findings of the mini EDHS were to the contrary. This lead the Tigray regional health bureau to call and initiate the present study so that to verify the findings of the mini EDHS for the region. However, studies addressing the proportion of women utilizing modern contraceptives and its associated factors are limited in the study area.

Further, determining the prevalence and associated factors in the actual local setting is important to take appropriate and tailored interventions. Therefore this study was aimed at determining the prevalence and associated factors of modern contraceptive utilization among married women of the reproductive age group in Edaga hamus town.

## Methodology

### Study setting

A community-based cross-sectional study was conducted from April 23 to May 10, 2017, at Edagahamus city, Tigray regional state of Ethiopia. Edagahamus is founded in the eastern zone of Tigray, wereda Saesie Tsaida Amba; which is located 885 Km north of the Ethiopian capital city of Addis Ababa, 105 Km east of the Tigray capital city Mekelle and around 20 Km near to Adigrat. Edagahamus is divided into four kebeles and the total population was 21,993; from those 10,031 were male and 11,962 were female. There is only one health center in Edagahamus and 3 private clinics.

### Participants

All women of reproductive age who reside in Edagahamus were taken as the study population. All women in the reproductive age group (15–49) are included, while women who were not mentally competent or who had any psychiatric disorders and critically ill during data collection were excluded.

### Sample size determination

By taking into consideration, 35.2% of the prevalence of modern contraceptives in Tigray region, EDHS 2016[6]. 95% confidence level, 5% tolerable margin of error, possible nonresponse rate of 10%, a total sample of 386 was taken. To check for the adequacy of the sample size, Epi info was used by considering factors associated with modern contraceptive use. By comparing sample size based on a single population proportion formula and Epi-info, the sample size determined by the single population proportion was greater than that of the Epi-info. Therefore the largest sample size of 383 was taken.

The required sample size calculated using the formula

$$\text{n}={\text{z}}_{\text{a}/2}2\text{pq}/\text{d}2,$$

Where n = sample size;

z = (1.96);

P = estimate of key proportion.

n = (1.96)2*0.352(1–0.352)/ (0.05*0.05) = 350.5~ 350.5 + 10% non response rate, the final n would be; 351+ 35 = 386

### Sampling procedure

The probability sampling technique was employed. Edagahamus is divided into four kebeles then, the sample size was allocated to each selected kebeles proportionally based on their expected number of women in reproductive age in each kebeles. The study participant was selected by systematic random sampling method for the households every 8^th^ household.

### Study variables

#### Dependent variables

Modern contraceptive utilization.

#### Independent variables

Socio-demographic and economic variables, Reproductive history, Socio-psychological factors, Source of information, Knowledge, and Attitude of modern contraceptive.

### Operational definition

**Modern contraceptive methods**: Including injectables, pills, implants, intrauterine contraceptive devices (IUCD), condoms, tubal ligation, and vasectomy.

**Utilization**: Using any of the above modern contraceptive methods to space the child and to protect unwanted pregnancy. **Current use**:—A woman who is using a modern contraceptive method at the time of the study. **Ever user**:—A woman who has practiced modern contraceptive methods sometime in the past but not using at the time of this study.

**Knowledge of modern contraceptive methods**:—According to this study if a woman mentions one of the modern contraceptive methods considers that she has good knowledge of modern contraceptive methods.

**The attitude of modern contraceptives**: was assessed by a Likert scale. Responses were dichotomized and summed. Having a positive response to at least 75% of statements was considered a positive attitude. Attitude statements included feelings towards the benefits of contraception (for both woman and family) and side effects.

**Keble**: A small administrative unite consisting of 20.000 population.

### Data collection tools and techniques

Data was collected by using an interviewer-administered and structured questionnaire adapted from different similar research with modification according to the context of the study area. To establish face validity and translation quality the questionnaire was tested on 38 women in reproductive age in a similar village population from selected adjacent kebeles in the district by data collectors and supervisors during training. A few questions, language clarity and information were revised and the questionnaire was finalized for the study. The questionnaire includes socio-demographic, economic status, Reproductive history, Socio-psychological factors, Source of information and Knowledge of modern contraceptives.

### Data quality assurance and control

Five health professional data collectors and two supervisors were recruited from the Health Center and they were given training for one day. The supervisors followed the process of data collection daily, checked the data completeness consistency and communicate with principal investigators daily.

### Data processing and analysis

Data was coded, cleaned, recorded and entered Epi info 7and finally export to SPSS version 22.00 for analysis. Simple descriptive summary statistics were done. Tables, statements, charts, and graphs were used to present the result of the analyzed data. Associations between independent and dependent variables were analyzed first using bivariate logistic regression analysis. Variables that had p<0.2 on bivariate analysis were entered multivariable logistic regression analysis. After checking using chi-square test variables with small cell size were merged into related categories. Appropriate model diagnostics and goodness of fit tests were done. Multicollinearity was checked to test correlation among predictor variables and Hosmer and Lemeshow test P-value (>0.2) were conducted to see model fitness. The statistical association between the different independent variables about dependent was measured using OR, AOR, 95% CI and P-values <0.05 was considered statistically significant.

### Ethical approval and consent to participate

Ethical clearance was obtained from the Ethical Review Board of Adigrat University, College of Medicine and Health Sciences and it is also got granted from the Health office of Adigrat hospital. Verbal and written consents were obtained after explaining their full right to refuse, withdraw any time, without any explaining or giving reasons. Information's obtained from individuals’ participants was kept secure and confidential. Names and other identifying data of respondents were made by using code throughout the study process to obtain confidentiality. Finally, data were collected according to the standard questionnaire prepared.

## Results

### Socio-demographic characteristics

A total of 383 Reproductive age group women participated in a response rate of 100%. Out of the total participated women, 64 (16.7%) were with an age range of 15–19 years. Nearly half of 163 (42.6%) participants were housewives. (Table 1, Figs 1, 2 and 3).

**Table 1:** Characteristics of participants in the study of contraceptive utilization at Edagahamus, northern Ethiopia, 2017.

Socio- demographic and economic factors	Frequency	Percent (%)
**Age**		
15–19	55	14.4
20–24	96	25.1
25–29	80	20.9
30–34	83	21.7
35–39	23	6.0
40–44	34	8.9
45–49	12	3.1
**Ethnicity**		
Tigray	344	89.9
Afar	35	9.1
Amhara	4	1
**Religion**		
Orthodox	329	85.9
Muslim	48	12.5
Protestant	3	0.8
Catholic	3	0.8
**Occupational status**		
Housewife	163	42.6
Merchant	129	33.7
Governmental employee	28	7.3
Student	40	10.4
Farmer	2	0.5
daily labor	21	5.5

**Fig 1:** Educational status of women in reproductive age.

**Fig 2:** Educational status of husband.

**Fig 3:** Marital status of women of reproductive age.

### Reproductive characteristics

Nearly three fourth of the respondents (74.4%) reported that they had a pregnancy. Among them, 96.1% of these pregnancies were wanted. Most of the respondents (46.5%) had 1–2 live births, 81 (28.9%) had 3–4 live birth and 70 (24.6%) had 5 and above live birth. One hundred seventy-seven (30.54%) of women respond it could be that too many children can improve family income. (Table 2).

**Table 2:** Characteristics of participants in the study of contraceptive utilization at Edagahamus, northern Ethiopia, 2017.

Reproductive factor	Frequency	Percent (%)
**Having any pregnancy before**		
Yes	285	74.4
No	98	25.6
Were pregnancy wanted		
Yes	274	96.1
No	11	3.9
**No. of live births**		
1–2	132	46.5
3–4	81	28.9
5 and above	70	24.6
**No. Of living children**		
1–2	130	46.1
3–4	90	31.9
5 and above	62	22
**History of abortion**		
Yes	74	26
No	211	74
**Type of abortion**		
Induced	11	14.9
Spontaneous	63	85.1
**Respondents age at first pregnancy**:		
<18	113	39.6
18 and above	172	60.4
**Children desired to you have**		
1–3	34	8.9
4–5	212	55.4
6 and above	137	35.8
**Having too many children help to improve the income of the family**		
Yes	117	30.5
No	266	69.5
**Having too many children guarantee generational continuity**		
Yes	173	45.2
No	210	54.8
**Should child mortality have compensated by too much birth**		
Yes	128	33.4
No	255	66.6
Is it a sin to practice MC method		
Yes	138	36
No	245	64
Does child spacing help to the health of the mother and child		
Yes	342	89.3
No	41	10.7
MC has side effect will be it dangerous to the mother		
Yes	188	49.1
No	191	49.9
I do not know	4	1
Does contraceptive use decrease sexual satisfaction		
Yes	69	18
No	272	71
I do not know	42	11
Does contraceptive cause infertility in women		
Yes	136	35.5
No	221	57.7
I do not know	26	6.8
Should men share responsible for FP use		
Yes	282	73.6
No	101	26.4

### Knowledge on modern contraceptive

In our study, all respondents heard about modern contraceptives. Among all respondents, most of the information about contraceptives got from health institution i.e. 220.199, 183, 48,176 of the respondents also get the information from radio, television, newspaper, and friend (neighborhood) respectively. About knowledge the different types of modern contraceptive 345 of the respondents knew pills, 364 knew injectable, 261 knew implant, 199 knew condom, 173 knew IUCD. Generally, 73.6% of the respondents had good knowledge while the rest were poor. Regarding number 58(15.2%) of respondents knew with the interval of 1–2, 223(58.2) knew from 3–4 number of contraceptives and 102(26.6%) knew 5 and above (Table 3, Fig 4).

**Table 3:** Knowledge of participants in the study of modern contraceptive utilization at Edagahamus, northern Ethiopia, 2017.

Variables	Frequency	Percent (%)
Have you heard about contraceptive		
Yes	383	100
No	0	0.0
**Source of information**		
Radio	199	52%
Television	183	47.8%
Newspaper	48	12.5
Health institution	220	57.4
Friend (neighborhood)	176	46%
Types of contraceptive you know		
Pill	345	90.1%
Injectable	364	95%
Implant	261	68.1%
IUCD	173	
Condom	199	52%
How many MC do you know		
1–2	58	15.2
3–4	223	58.2
5 and above	102	26.6

**Fig 4:** The source of contraceptive.

### Attitude of women towards using modern contraceptives

As regards to attitude of women on using modern contraceptive two hundred forte three (63.4%) of respondents had a positive attitude respectively. Among non-users the reason included where fear of side effect (4.4%), disagreement with the husband (2.5%), religious reason (3.2%), community reason(0.6%) and other(89.3%)(separation). In our study among the participants, 254(66.3%) of the participants were respond that yes for cultural acceptance of the utilize of modern contraceptives by the community and 129(33.7%) of them respond no for cultural acceptance. (Table 4)

**Table 4:** Attitude of women towards using modern contraceptives at Edagahamus, northern Ethiopia, 2017.

Variables	Frequency	Percent (%)
**Do you use any method of MC**		
Yes	224	58.5
No	159	41.5
**If no why**		
Fear of side effect	7	4.4
Disagreement with husband	4	2.5
Religious reasons	5	3.2
Community reason	1	0.6
Other	142	89.3
Cultural acceptance		
Yes	254	66.3
No	129	33.7
Religious fathers' acceptance		
Yes	13	3.4
No	370	96.6
Feeling of husband		
Positive	151	62.1
Negative	42	17.3
Nothing	50	20.6
Communication with husband MC		
Sometimes	76	30.4
Always	107	42.8
No communication	67	26.8
Weakness observed so far		
shortage of contraceptive	2	0.9
shortage of health professional	4	1.8
poor client approach	17	7.5
no weakness	203	89.8

### Modern contraceptive utilization

Overall prevalence of modern contraceptive utilization in Edagahamus town was found to be two (58.5%). Majority of the contraceptive ever used 121 (54.4%) use injectable contraceptive methods followed by pills 33 (14,7) and implants 31 (13.5%) respectively. (Figs 5 and 6).

**Fig 5:** Type of contraceptive ever used.

**Fig 6:** Currently used contraceptive.

### Factors affecting modern contraceptive utilization among reproductive women

Age, Educational status of the husband, Number of children wanted and Communication with the husband of MC have significantly associated with modern contraceptives in Edagahamus. Women in the age group of 25–29 years were 59.4% (AOR = 0.406; C1 = 0.000, 0.398; P = .017) times less likely to use modern contraceptives as compared to those age group of 15–19 years. The odds of the utilization of modern contraceptives in the study area were 86.5% times (AOR = 0.135; 95% C1 = 0.002, 0.760; P = .033) less likely to use MC among 30–34 years as compared to women of 15–19 Years of age.

The odds of the utilization of modern contraceptive among education status of an illiterate husband were 99.7% times less likely to use than whose educational status 9–12 (AOR = 0.003;95%CI = 0.000,0.316;P = 0.014*) and Illiterate were 99.6% less to use than diploma and above(AOR = 0.004;95%CI = 0.000,0.631;P = 0.032). However, women who want to have number of children 1–3 were 10.8 times more likely to used modern contraceptive than who want 6 and above children (AOR = 10.802; 95%CI; 4.027, 28.975;P = 0.000) and women who want to have 4–5 were 3 times more likely to practice modern contraceptive than who want to have 6 and above (AOR = 2.624;95%CI = 1.437,4.791;P = 0.002).

A woman whose husband who had a negative feeling towards the utilization of modern contraceptive was 0.814 times less likely to use modern contraceptive than who had a positive feeling (AOR = 0.186;95%CI = 0.056,0.617; P = 0.006) (Table 5).

**Table 5:** Bi variable and multivariable logistic regression model for factors associated with contraceptive utilization at Edagahamus, northern Ethiopia, 2017.

Variable	Modern contraceptive use		COR (95% CI)	AOR
	yes	no		
**Age in years**				
15–19	9	46	1	1
20–24	66	30	0.089, (0.039,0.205)*	0.055(0.003,1.081)
25–29	77	3	0.008(0.002,0.03)*	0.406(0.000,0.398)*
30–34	59	24	1.152(0.21,0.133)	0.135(0.002,0.760)*
35–39	9	14	0.210(0.92,0.481)	0.069(0.002,2.591)
40–44	2	32	0.250(0.98,0.639)	1.575(0.000,6.693)
45–49	2	10	0.667(0.177,2.513)	0.742(0.003,17.124)
**Educational status**				
Illiterate	5	30	1	1
Can read write	2	3	0.250(0.033,1.893)*	0.681(0.000,5.995)
1–4	17	6	0.059(0.016,0.222)*	0.52(0.14,17.984)
5–8	31	30	0.161(0.161,0.056)*	0.293(0.008,10.443)
9–12	81	76	0.156(0.058,0.424)*	0.822(0.021,31.926)
Diploma and above	88	14	0.027(0.009,0.080)*	0.901(0.340,4.107)
**Educational status of husband**				
Illiterate	5	35	1	1
Can read and write	2	20	1.389(0.247,7.823)	5.702(0.569,5.709)
1–4	8	15	0.089(0.025,0.313)*	1.767(0.67,39.845)
5–8	49	13	0.045(0.015,0.136)*	0.074(0.003,1.949)
9–12	54	7	0.025(0.008,0.081)*	0.003(0.000,0.316)*
Diploma and above	63	2	0.005(0.001,0.025)*	0.004(0.000,0.631)*
**Marital status**				
Unmarried	24	105	1	1
Married	179	24	0.032(0.008,0.124)*	0.000(0.000,)0.999
Divorced	18	22	1.193(0.309,4.609)	0.000(0.000,)0.999
Widowed	3	11	0.333(0.081,1.380)*	0.000(0.000,)0.999
**Occupational status**				
Housewife	100	63	1	1
Merchant	87	42	0.766(0.472,1.244)	0.348(0.054,2.228)
Government employee	21	8	0.605(0.523,1.448)	2.682(0.029,24.796)
Student	6	34	8.995(3.572,22.647)*	2.950(0.000,9.838)
Daily labor	10	12	1.905(0.777,4.668)*	0.007(0.000,3.180)
**Income**				
<600	99	97	1	1
600–1200	61	42	0.703(0.434, 1.139 )*	0.127(0.011, 1.523)
>1200	64	20	0.319(0.1790.567,) *	0.595(0.072,4.938)
**Have any pregnancy**				
Yes	190	95	1	1
No	34	64	3.765(2.322,6.105) *	0.852(0.090,8.046)
**Number of pregnancies**				
1–2	76	47	1	1
3–4	58	25	0.697(0.385,1.262)	0.797(0.423,1.501)
5 and above	56	21	0.664(0.362,1.218)*	1.191(0.590,2.402)
**Number of children wanted**				
1–3	16	18	10.362(4.661,22.088)*	10.8(4.027,28.975)*
4–5	116	96	3.910(2.430,6.318)*	2.624(1.437,4.791)*
6 and above	92	45	1	1
**Feeling of the husband towards MC**				
Negative	40	64	1	1
Positive	163	26	0.036(0.013,0.095)*	0.186(0.056,0.617)*
Nothing	48	**42**	1.145(0.456,2.876)	0.036(0.005,1.233)
**Communication with the husband of MC**				
Sometimes	90	36	0.113(0.053,0.243)*	0.300(0.070,1,288)
Always	125	23	0.008(0.002,0.036)*	3.176(0.894,11.279)
No communication	40	69	1	1

Note: *-significant results, 1-reference category **p-value<0.001, *p-value≤0.05

## Discussions

This study was conducted to assess the Prevalence and determinants of modern contraceptive utilization among Women in the Reproductive Age Group in Edaga-hamus Town, Eastern zone, Tigray Region, Ethiopia. In this study, the current prevalence of modern contraceptive utilization was 58.5%. The result is in line with the study conduct in Addis Abeba (56.3%) and Lusaka, Zambia (59.2%) [6, 14, 19]. The variations may be due to different population characteristics. However, the prevalence of modern contraceptive utilization in this study was higher than the study conduct in Ofla District, Tigray, Northern Ethiopia (37.1%) [10], in Tigray, North Ethiopia(35.6%) [11], in Humera town, Tigray Region, Ethiopia(27.1%) [12], in Tigray, Ethiopia(46%) [13], in South Nigeria (21.6%) [20]. United Nations millennium development goal (MDG) 2015 report for African continent (33.4%) [2], and the 2015 sub-Saharan MDG reports [2]. 2016 Ethiopian DHS for Amhara region, 46.9% [9], Gondar, Nekemte [21], Debreberhan [15], and west Gojjam [22], Ghana [22, 23], Kenya [2] and Nepal [24]. The United Nations MDG 2015 report for Somalia, Eritrea, and South Sudan which was 23.7, 20 and 6.8% respectively [2]. This difference might be because of socio-demographic and cultural variation. Besides, there is a difference in the study time interval between other studies done and this study. Moreover, the discrepancy may be due to an educational grade of study participants, up-to-date house to house health education policy by HEW more organized in the town through the Ethiopian federal ministry of health. However, this result is lower than the results in Benin City, Nigeria (64.5%) [25], Holeta town (73%) [5], Mbarara, Uganda (85%)%) [26], and Lesotho (82–86%)%) [26, 27], respectively. This discrepancy might be due to the age difference or and religion of the participant and the other reason might be due to geographical variation. The commonest modern contraceptive method utilizing by up-to-date married men wife was injectables (54.4%), pills (14.7%) and implants (13.5%) married men were male condoms (2.2%) this is similar with study conduct in Holeta town [5], (injectable 48% followed by implant 15.3% and pill 5.4%. This showed they were aware of family planning and they knew the different methods. This study revealed that the odds of those age 15–19 years were less likely to use modern contraceptives by 59.4% and 86.5% as compared to age 25–29 and 30–34 years. This study similar to study conduct in Ethiopia demographic and health survey, 2016 [6] and contrary with study conduct in shire Endaslasie [28]. This may be due to those who are 15–19 where most of them were unmarried but those 25–29, 30–34 were most of them are married and within this range of age, their educational status was high. Mother who had negative husband approval towards modern contraceptive utilization were 81% less likely to use MC than who approve it positive husband approval. This finding of the study was supported by study conduct in Farta district south Gondar in 2014 [29]. This might be due to the educational status of husbands who had high educational status were good approval towards modern contraceptives. The odds of the utilization of modern contraceptive among education status of an illiterate husband were 99.7% times less likely to use than whose educational status 9–12 (AOR = 0.003;95%CI = 0.000,0.316;P = 0.014*) and Illiterate were 99.6% less to use than diploma and above (AOR = 0.004;95%CI = 0.000,0.631;P = 0.032). This agreed with the studies conducted in most developing countries [17, 21, 22]. This can be explained by the notion that women with better educational levels have better access to health care information, have greater autonomy to make decisions and have a greater ability to use quality health care services [30, 31]. In this study mother who went to have several children, 1–3 and 4–5 were eleven and three times more likely to used modern contraceptive than who went 6 and above children. It might be to attain their desired number of children and the spacing and timing of their births. This finding is similar to previous reports from Zambia, Northwest Tigray and Uganda which reported that as the number of living children increases, the use of modern contraceptive increases [15, 19, 26].

## Limitation

Since this study was limited to married women only at the time of the study; results may not be generalized to all women in Edagahamus town.

The study design is cross-sectional; therefore it may be difficult to establish a temporal relationship.

## Conclusion and recommendation

Modern contraceptive utilization was still low (far below the national target). Factors such as age, educational status of the husband, the number of children wanted and feeling of the husband was associated with the utilization of modern contraceptive. Therefore, train health professionals especially health extension workers to raise awareness education, enhance information, education and communication activities regarding modern contraceptives and create awareness about the quality of life and healthy live hood to the community through the training of health professionals to convince the community.

## Supporting information

S1 File Questionnaire English version. (DOCX)

S2 File Questionnaire in local language. (DOCX)

S3 File Data set. (SAV)

## Abbreviations

ADU: Adigrat university
C.I: Confidence Interval
CMR: Child mortality rate
CPR: Contraceptive Prevalence Rate
DHS: Demographic and Health Survey
HIV: Human immune virus
IPPF: International Planned Parenthood Federation
IUCDs: Intra-Uterine Contraceptive Devices
LAM: lactation amenorrhea method
MC: Modern Contraception
OCP: Oral Contraceptive Pill
SDM: standard days method
TFR: Total Fertility Rate
WHO: World health organization
